The article "Evaluating the spillover effects of the Sugira Muryango home-visiting intervention on temperament of children aged (0.3–3years) exposed to domestic violence: A cluster randomized controlled trial" was retracted in 2025. Reasons: errors in the data; errors in the analysis; no approval from an author; no approval from a third party.

# Evaluating the spillover effects of the Sugira Muryango home-visiting intervention on temperament of children aged (0.3–3years) exposed to domestic violence: A cluster randomized controlled trial

**DOI:** 10.1371/journal.pone.0320595

**Published:** 2025-03-31

**Authors:** Theodat Siboyintore, Jeanne Marie Ntete, Jean Mutabaruka, Theresa Betancourt, Sarah Jensen, Vincent Sezibera

**Affiliations:** 1 Department of Psychiatry and Behavioral Sciences, College of Medicine and Health Sciences, University of Rwanda, Kigali, Rwanda; 2 Boston College School of Social Work, Boston College, Chestnut Hill, Massachusetts, United States of America; 3 Centre for Mental Health, College of Medicine and Health Sciences, University of Rwanda, Kigali, Rwanda; IFPRI: International Food Policy Research Institute, United States of America

## Abstract

**Background:**

Domestic violence, intimate partner violence, and violence against children and women adversely affect children’s well-being. The Sugira Muryango Program (SM) in Rwanda, a home-visiting intervention, aimed to to improve caregiving practices and family dynamics, may also have potential indirect effects on children’s temperament.

**Objectives:**

This study assesses the impact of SM on the temperament of younger children whose families benefited from the intervention, comparing their temperament with those under usual care.

**Methods:**

This study utilized a spillover effect cohort design, focusing on 247 younger siblings of children enrolled in the Sugira Muryango Program (SM) to assess potential spillover effects of the intervention. The temperament of these siblings was measured using the Infant Behavior Questionnaire–Revised Short Form, which was translated into native language of the respondents. Multiple linear regression analysis was performed using SPSS version 29, with the treatment group (SM vs. UC) as the main predictor and temperament as the dependent variable.

**Results:**

The analysis showed no statistically significant differences in key temperament traits such as surgency, negative emotionality, and orienting capacity between the intervention and control groups. The findings indicated that changes in surgency (B =  1.984, t =  1.183, p =  0.24), negative emotionality (B =  -1.657, t =  -0.915, p =  0.36), and orienting capacity (B =  0.551, t =  0.313, p =  0.75) were not significant.

**Conclusion:**

The results suggest that SM had limited spillover effects on the temperament traits of younger siblings. Given that the intervention was primarily designed to improve broader family dynamics rather than directly impact child temperament, these findings highlight the importance of focusing on direct intervention strategies aimed explicitly at the target child population. Future research should align with the theory of change by examining caregiver-related outcomes, such as parenting practices and mental health, which may influence child temperament. Additionally, considering potential external factors like the COVID-19 pandemic may have influenced the effectiveness of the intervention.

The article "Evaluating the spillover effects of the Sugira Muryango home-visiting intervention on temperament of children aged (0.3–3years) exposed to domestic violence: A cluster randomized controlled trial" was retracted in 2025. Reasons: errors in the data; errors in the analysis; no approval from an author; no approval from a third party.

## Background

Globally, more than one billion children, over half of the world’s child population, experience physical, emotional, or sexual violence annually, underscoring the urgent need for interventions [1,2]. Violence against children (VAC) includes domestic violence, neglect, maltreatment, and exploitation, and is often compounded by exposure to parental intimate partner violence (IPV), which creates overlapping impacts within families [3]. Children exposed to IPV face an increased risk of direct physical violence, which can lead to significant mental health challenges and developmental delays [4]. The co-occurrence of VAC and IPV is driven by shared risk factors, including caregiver stress, poor mental health, economic hardship, and rigid gender norms, which exacerbate their consequences and increase vulnerability [5,6]. These factors exacerbate the consequences of violence and increase children’s vulnerability.

In Rwanda, the first national population-based survey on violence in children and youth aged 13 to 24 was conducted in 2015 [7]. The survey revealed that 50% of females and 65% of males had experienced some form of violence before turning 18 years, with notable gender disparities. Boys were more likely to experience physical violence (59.5% versus 37.2%) and emotional violence (17.3% versus 11.2%), while girls were more likely to experience sexual violence (23.9% versus 9.6%)2 [7]. Additionally, a study by Jensen [4] found that 43% of Rwandan parents use violent discipline, and 27% of female caregivers report IPV victimization among socioeconomically vulnerable families with children aged 6 to 36 months in rural settings [4,8]. Furthermore, data from the 2019/20 Demographic and Health Survey (DHS) highlights rising IPV rates among women compared to the 2014/15 DHS (from 40% in 2015 to 46% in 2020), underscoring the escalating trends in violence [8,9]. These findings highlight the interconnected nature of VAC and IPV, emphasizing the need for holistic interventions that address both forms of violence simultaneously.

The consequences of children witnessing parental family violence are profound. Meta-analyses of 118 studies show that approximately 63% exhibit poor health outcomes [10]. In Rwanda, a study involving 548 participants found that children exposed to IPV were more likely to develop mental health issues such as depression, anxiety, and irritability [11]. These children frequently report higher mood fluctuations, as well as feelings of dread, despair, anger, and frustration, as well as low self-esteem [5,12–14]. The extent and duration of these adverse effects are intricately linked to the nature of the problems and the availability of protective factors.

The article "Evaluating the spillover effects of the Sugira Muryango home-visiting intervention on temperament of children aged (0.3–3years) exposed to domestic violence: A cluster randomized controlled trial" was retracted in 2025. Reasons: errors in the data; errors in the analysis; no approval from an author; no approval from a third party.

Recognizing the urgency to counter childhood abuse, global initiatives, including the INSPIRE technical package, have been instrumental in providing evidence-based strategies to prevent and respond to violence against children [3,15]. In Rwanda, innovative interventions such as the Vision 2020 Umurenge Programme and the Sugira Muryango (SM) intervention have been implemented to combat family violence and enhance early childhood development [16]. Vision 2020 Umurenge Programme, a social protection program, provides direct assistance to low-income families with young children, while the SM intervention employs community-based approaches.

The SM intervention, implemented from June to September of 2018, involved 12 weekly modules delivered by trained community coaches [6]. These modules focused on positive parenting, stress management, nutrition and hygiene practices, and conflict resolution. Eligible families were those with young children facing vulnerabilities such as poverty and limited access to resources. The intervention was delivered by community coaches—trained volunteers with a background in child and family support—who tailored the program to meet the unique needs of each family.

Grounded in evidence-based strategies from the Nurturing Care Framework and UNICEF/World Health Organization’s Care for Child Development, the SM ntervention aimed to foster positive parenting practices, reduce harsh disciplinary methods, and improve family dynamics. Its impacts are notable: a recent sudy showed that immediately post-intervention, the odds of exposure to harsh discipline decreased by 70%, and the odds of female caregivers reporting IPV victimization decreased by 51% in SM families compared to control families [17]. Additionally, other study has found that SM have succeeded in creating a healthy, stimulating, and safe environment that supports children’s achievement of developmental milestones [6].

Temperament, defined as an individual’s innate behavioural and emotional traits, plays a critical role in how children interact with their environment, build interpersonal relationships, and navigate challenges [18]. It evolves over time, shaped by both genetic predispositions and environmental experiences [19,20]. Temperament is closely linked to various developmental outcomes, including emotional regulation, social competence, and cognitive functioning. Children with more adaptive temperaments are better equipped to thrive in nurturing environments, while those with more challenging temperaments may require additional support to reach their developmental potential.

The article "Evaluating the spillover effects of the Sugira Muryango home-visiting intervention on temperament of children aged (0.3–3years) exposed to domestic violence: A cluster randomized controlled trial" was retracted in 2025. Reasons: errors in the data; errors in the analysis; no approval from an author; no approval from a third party.

Although the SM intervention was not explicitly designed to directly impact child temperament, it can be argued that its focus on improving caregiver practices and family dynamics has significant spillover effects on temperament and overall child development. This study evaluated these potential spillover effects, hypothesizing that toddlers in families benefiting from the SM intervention would exhibit improved temperament compared to those receiving usual care (UC). Furthermore, this research aims to contribute to the understanding of how programmatic interventions can influence child temperament, thereby supporting broader discussions on effective mental health strategies within the SM Program context.

## Methodology

### Research design and setting

This study employed a spillover effect cohort design to examine the indirect effects of the Sugira Muryango (SM) intervention on younger siblings in rural Rwandan families. Conducted from January 21, 2022, to January 2023, it targeted families from lower socioeconomic backgrounds (Ubudehe categories) in the rural districts of Ngoma, Nyanza, and Rubavu. In the original cluster-randomized controlled trial (CRCT), which focused on direct effects, families were randomly assigned to intervention or control groups. This study focused on younger siblings who did not directly receive the intervention, using validated temperament measure to assess potential spillover effects.

### Participants

The quantitative component of the main trial initially involved approximately 1084 children and 1498 caregivers and intimate partners [6]. This follow-up study focused on a subset of 247 young children who were not directly involved in the original program but belonged to families that participated in the main trial implemented in 2018–2019. Families were selected from both the intervention (Sugira Muryango) and control (Usual Care) groups to allow for comparative analysis of spillover effects.

Eligibility criteria required that younger siblings (a) be aged between 3 months and 3 years old at the time of data collection and (b) have a caregiver who participated in the main trial with a documented history of domestic violence. Toddlers (aged 3 months to 3 years) were selected as the target group due to their critical developmental stage, during which environmental influences, including caregiving practices, significantly shape temperament and developmental outcomes [21].

The article "Evaluating the spillover effects of the Sugira Muryango home-visiting intervention on temperament of children aged (0.3–3years) exposed to domestic violence: A cluster randomized controlled trial" was retracted in 2025. Reasons: errors in the data; errors in the analysis; no approval from an author; no approval from a third party.

To avoid clustering of data at the household level, only one young sibling per household was included. If multiple children met the criteria within a household, one child was randomly selected using an excel-based randomization (=RAND()) to ensure unbiased sampling. Recruitment for this study took place from January to May 15, 2022, and data were collected at a single time point, approximately four years after the intervention, to assess long-term spillover effects.

Since the sample size was determined by the availability of eligible children within participating families, this study utilized a convenience sampling method. Unlike the main trial, no power analysis was conducted specifically for this subset, as not all families had children aged 3 months to 3 years at the time of data collection. No eligible participants declined to participate, as this study relied on families already involved in the main trial, ensuring full retention of the available sample. The final sample size comprised 247 children, split into 122 in the control group and 125 in the treatment group.

### Procedures

The spillover study builds on the original Sugira Muryango (SM) trial, which was registered as a cluster-randomized controlled trial (registration number NCT02510313). This registration was updated to include the spillover study to assess the long-term impacts of the intervention on younger siblings. Ethical approval for this spillover study was obtained from the Rwanda National Ethics Committee (No. 15/RNEC/2022).

Since the study involved children aged 3 months to 3 years, informed consent was obtained exclusively from the mothers of participating children, who were the primary caregivers and the sole providers of data. Given the developmental stage of the children, obtaining assent was not applicable. This approach was fully compliant with ethical guidelines, as approved by the ethics committee.

Before data collection, all study tools were professionally translated into Kinyarwanda and back-translated to ensure linguistic and cultural relevance. The tools were specifically designed to facilitate accurate and reliable responses from mothers regarding the temperament and caregiving environment of their children.

A team of enumerators were recruited and underwent comprehensive training prior to data collection. The training included modules on ethical research practices, the objectives of the evaluation, the content of the questionnaire, and the use of the Kobo data collection tool. Enumerators were also trained in qualitative interviewing techniques and received specific instruction on the SM intervention to enhance their understanding of the study context. This rigorous preparation ensured high-quality data collection while upholding the ethical standards of research.

The article "Evaluating the spillover effects of the Sugira Muryango home-visiting intervention on temperament of children aged (0.3–3years) exposed to domestic violence: A cluster randomized controlled trial" was retracted in 2025. Reasons: errors in the data; errors in the analysis; no approval from an author; no approval from a third party.

### Study tools

#### Sociodemographic information.

Sociodemographic data were collected on district (Ngoma, Nyanza, Rubavu), child gender (male or female), and age (0–17 months, 18–37 months, 38–53 months) to account for developmental and contextual differences. Caregivers also reported their participation in other parenting programs (Yes or No) to control for external influences.

#### The infant behaviour questionnaire–revised short form.

The IBQ– RSF is designed to measure three broad factors of infant temperament: negative emotionality (NEG); positive affectivity/surgency (PAS) orienting capacity (OC) [22]. There are 37 questions in total, and each one asks parents to report how often their baby behaved in a particular way over the last 7 days. The items were rated on using 8 points-Likert scale ranging from 1 (does not apply), to 8 (always), [22]. Items rated as 1 was treated as missing. This questionnaire was administered to the young siblings aged from 3 months to 3 years old.

### Intervention component

As stated earlier in introduction, the Sugira Muryango (SM) intervention was conducted between May 7 and September 14, 2018, beginning within two weeks of baseline data collection, and staggered across districts to allow for efficient implementation. Designed as a home-visiting program, the intervention employed trained community coaches to deliver 12 weekly sessions focused on enhancing responsive caregiving, improving family nutrition and hygiene, and reducing harsh disciplinary practices*.* Fig 1 represents the Theory of Change, illustrating the hypothesized long-term outcomes of the intervention. The 4-year post-intervention outcomes included in the figure are theoretical expectations based on the program’s objectives and prior evidence, not direct results from this spillover study.

**Fig 1:** Theory of change.

Community coaches provided tailored psychoeducation to families, engaging both male and female caregivers in activities aimed at improving household dynamics and child well-being. Each visit included a 15-minute active play session during which caregivers received real-time feedback on parent-child interactions [23], emphasizing the importance of responsive caregiving and active engagement. Families were also supported in accessing formal resources, such as government programs for health and nutrition, and informal supports like neighbors and extended family networks to address specific challenges, including housing insecurity and food scarcity.

The article "Evaluating the spillover effects of the Sugira Muryango home-visiting intervention on temperament of children aged (0.3–3years) exposed to domestic violence: A cluster randomized controlled trial" was retracted in 2025. Reasons: errors in the data; errors in the analysis; no approval from an author; no approval from a third party.

The intervention drew upon evidence-based frameworks, including the UNICEF/WHO Care for Child Development package [24] and Nurturing Care Framework, emphasizing holistic family support. Although the primary aim was to improve caregiver behaviors and family dynamics, these changes were hypothesized to have indirect spillover effects on the temperament of younger children in the household. By tailoring the program to meet the unique needs of each family, the SM intervention demonstrated its potential as a scalable model for promoting early childhood development in resource-constrained settings.

### Data analysis

For quantitative methods, the analyses were carried out in SPSS version 29 by fitting a multiple linear regression (OLS) model for continuous outcomes with treatment group (SM vs UC) as the main predictor, whereas temperament subscales as dependent variable [6]. Considering the very low intra-class correlation and small sample size, layer of nesting such as randomization clusters or regions were not considered. In the OLS model, we controlled covariates such as age, gender, and participation in other parenting programs. Under intention-to-treat assumptions, we replaced lost cases using multiple imputation [25]. We conducted sensitivity analyses to evaluate the impact of imputation on our results. The amount of missing data was minimal, with less than 5% of cases requiring imputation. To evaluate the effects size (Cohen’s d) of the intervention between the groups, we computed independent t-test. Significance was considered observed at p = 0.05 (two tailed).

## Results presentation

### Sociodemographic characteristics of study participants

The study included 247 children divide into two groups: 122 in the control group and 125 in the treatment group (Table 1). Rubavu had the highest representation, with 45 children in the control group and 47 in the treatment group, while Ngoma had the smallest, with 41 participants in each group. The gender distribution showed a slight male predominance, with 56.6% boys in the control and and 52.0% in the treatment group. Age distribution also differed, with the control group having more younger children (36.1% aged 0–17 months) and the treatment group concentrated in the 18–37 months (48.0%).

**Table 1:** Sociodemographic characteristics (N = 247).

		Control (UC) (N = 122)	Treatment (SM) (N = 125)	p-value
		Frequency (%)	Frequency (%)	
District	Nyanza	36 (29.5)	37 (29.6)	P < 0.001
	Rubavu	45 (36.9)	47 (37.6)	
	Ngoma	41 (33.6)	41 (37.6)	
Child gender	Male	69 (56.6)	65 (52.0)	P < 0.001
	Female	53 (43.4)	60 (48.0)	
Age	[0–17] months old	44 (36.1)	33 (26.4)	P < 0.001
	[18–37] months old	39 (32.0)	60 (48.0)	
	[38–53] months old	39 (32.0)	32 (25.6)	
Participation in other programs	Yes	22 (18)	16 (12.8)	P < 0.001
	No	100 (82)	109 (87.2)	

Futhermore, the independent t-test showed no statistically significant differences between the treatment group (Sugira Muryango) and the control group (Care as Usual) across all temperament measures, including total temperament scores (mean difference (MD) =  −2.058, p =  0.66), surgency (MD = −2.383, p =  0.19), negative emotionality (MD =  1.700, p =  0.32), and orienting subscales (MD =  −1.375, p =  0.44), (Table 2). While the treatment group demonstrated slightly higher scores in surgency and orienting subscales, and the control group showed marginally higher scores in negative emotionality, these differences were not statistically significant.

The article "Evaluating the spillover effects of the Sugira Muryango home-visiting intervention on temperament of children aged (0.3–3years) exposed to domestic violence: A cluster randomized controlled trial" was retracted in 2025. Reasons: errors in the data; errors in the analysis; no approval from an author; no approval from a third party.

**Table 2:** Independent t-test analysis.

Treatment group (SM vs CAU)		Mean (SD)	Mean difference	P-value	Lower Confidence Interval	Upper Confidence Interval
Ibq_TOTAL scores	Control	79.04(18.01)	−2.058	P = 0.66	−11.58	7.47
	Treatment	81.10 (12.04)				
Surgency subscale	Control	24.16 (6.58)	−2.383	P = 0.19	−6.062	1.295
	Treatment	26.55 (5.26)				
Negative emotional subscale	Control	26.00(6.54)	1.700	P = 0.32	−1.83	5.233
	Treatment	24.30 (4.69)				
Orienting subscale	Control	28.87 (5.95)	−1.375	P = 0.44	−4.97	2.220
	Treatment	30.25 (5.80)				

### Effects of the Sugira Muryango intervention on temperament

To evaluate the potential spillover effects of the Sugira Muryango intervention on the temperament of younger siblings, our regression analyses incorporated controls for covariates such as age, gender, and participation in other parenting programs to control for potential confounding factors. Temperament outcomes were measured using the validated Infant Behavior Questionnaire (IBQ) (**Table 3**).

**Table 3:** Effects of the Sugira Muryango intervention on temperament among young siblings.

Outcome				
Child mental health and behaviors	B	s.e	t	Pvalue
**Surgency (IBQ)**	**1.984**	**1.677**	**1.183**	**0.244**
**Negative emotionality (IBQ)**	**−1.657**	**1.81**	**−0.915**	**0.366**
**Orienting capacity (IBQ)**	**0.551**	**1.758**	**0.313**	**0.756**
**Controlling variables: age, gender, other school program attendance**				

**Note: regression parameter refers to the treatment variable, 1 = treatment, 0 = Control)**

For **surgency**, which which reflects positive emotionality and activity levels, the analysis showed no statistically significant differences between the control and treatment groups (B =  1.984, p =  0.244). The size of the estimated effect suggests a small increase in positive emotionality among younger siblings in the treatment group, though it does not provide strong evidence for a spillover effect under the current conditions.

The article "Evaluating the spillover effects of the Sugira Muryango home-visiting intervention on temperament of children aged (0.3–3years) exposed to domestic violence: A cluster randomized controlled trial" was retracted in 2025. Reasons: errors in the data; errors in the analysis; no approval from an author; no approval from a third party.

For **negative emotionality**, encompassing feelings of anger and distress, although there was a reduction in these emotional responses, the effect did not reach statistical significance (B =  −1.657, p =  0.366). The size of the estimated effect suggests a small decrease in positive emotionality among younger siblings in the treatment group, though it does not provide strong evidence for a spillover effect under the current conditions.

Lastly, for orienting capacity, indicative of the child’s ability to focus attention and regulate emotional responses, the effects also did not reach statistical significance (B =  0.551, p =  0.75). This small effect size suggests minimal evidence of a spillover impact in this domain.

Overall, the findings indicate some directional trends, with slight increases in positive emotionality and attention regulation and a modest reduction in negative emotionality among younger siblings in the treatment group. However, these changes were not statistically significant, suggesting that, the Sugira Muryango program did not significantly influence the measured dimensions of temperament in younger siblings under the current study conditions.

## Discussion

Our study aimed to assess potential spillover effects of the Sugira Muryango (SM) home-visiting intervention on the temperament of younger siblings, who were not the intended beneficiaries of the original intervention implemented in 2018. The findings revealed no statistically significant differences across temperament dimensions, including surgency, negative emotionality, and orienting capacity between the treatment and control groups. These findings suggest that the intervention may not have produced significant spillover effects on child temperament. Several factors, including the design of the intervention, the time elapsed since implementation, and contextual influences may have contributed to these findings.

Our results align with findings from other home-visiting interventions that primarily target caregivers rather than children directly. Prior research has shown that while parenting programs can enhance caregiving behaviors and reduce harsh discipline, their indirect effects on child behaviour or temperament are often small or non-significant unless explicitly integrated into the intervention design [26,27]. For instance, a longitudinal study evaluating the Nurse-Family Partnership program in the U.S. found significant improvements in maternal parenting but limited effects on child emotional regulation [27]. Similarly, a study on the Parenting for Lifelong Health program in South Africa reported positive effects on parenting but no clear impact on child temperament [26]. These findings suggest that interventions primarily designed to modify caregiving practices may require additional components specifically addressing child emotion regulation and parent-child bonding to yield stronger temperament-related outcomes [28].

The article "Evaluating the spillover effects of the Sugira Muryango home-visiting intervention on temperament of children aged (0.3–3years) exposed to domestic violence: A cluster randomized controlled trial" was retracted in 2025. Reasons: errors in the data; errors in the analysis; no approval from an author; no approval from a third party.

It is essential to clarify that the SM intervention was delivered in 2018, well before the onset COVID-19 pandemic in the end of 2020. Therefore, the pandemic did not disrupt the design or implementation of the original program. While the 2022 data collection coincided with the pandemic’s aftermath, which could have influenced caregiving environment [29,30], both treatment and control groups were equally affected, making pandemic-related biases an unlikely explanation for the null findings. Instead, the study design itself offers a more plausible explanation. Unlike previous evaluations of SM that found reductions in harsh discipline and IPV, this study focused on younger siblings who were not direct intervention recipients. The absence of a direct intervention component targeting child temperament may explain the lack of significant spillover effects.

The time elapsed since the intervention also warrants consideration. Four years is a substantial period in early childhood development, during which a child’s temperament is influenced by many environmental and genetic factors [31]. Any early effects of the intervention may have faded, particularly if caregivers reverted to pre-intervention behaviors. This aligns with research indicating that the benefits of parenting interventions often diminish over time unless reinforced through booster sessions [32]. Sustained caregiver engagement and periodic reinforcement of positive parenting strategies may be necessary to maintain long-term effects on both caregiver behavior and child outcomes.

The study’s sampling methodology may also have influenced the results. The study utilized a convenience sample of younger siblings aged 3 months to 3 years from families involved in the original trial. While this approach allowed for the inclusion of all eligible children, the small sample size and age range may have limited the statistical power to detect subtle intervention effects. Additionally, caregiver-reported temperament measures, while widely validated and adapted to our context, its application in in this population may require further psychometric testing to ensure ensure cultural sensitivity and relevance. This is particularly important for accurately capturing the nuances in temperament that may be shaped by cultural practices and caregiving norms. Future studies should incorporate observational assessments or physiological measures of temperament to strengthen validity.

The article "Evaluating the spillover effects of the Sugira Muryango home-visiting intervention on temperament of children aged (0.3–3years) exposed to domestic violence: A cluster randomized controlled trial" was retracted in 2025. Reasons: errors in the data; errors in the analysis; no approval from an author; no approval from a third party.

## Strengths and limitations

This study contributes to the growing body of literature on the broader impacts of parenting interventions, offering valuable insights into the potential spillover effects of the SM program on younger siblings. However, the single time-point limits the ability to infer causality or observe longitudinal changes. Additionally, the study’s reliance on caregiver-reported data introduces potential biases, particularly under conditions of heightened stress, such as during or after the pandemic [29,30]. Future research should incorporate longitudinal designs, culturally adapted measurement tools, and objective measures of child temperament to strengthen the validity of findings.

## Conclusion

The evaluation of potential spillover effects of the SM intervention on younger siblings revealed no statistically significant differences in temperament dimensions, including surgency, negative emotionality, and orienting capacity. These findings suggest that while the intervention effectively improved caregiver behaviors, its indirect effects on child temperament were limited. Future research should explore the integration of explicit child-focused components in home-visiting programs, implement booster sessions to sustain long-term impacts, and utilize more objective measures of temperament to enhance the reliability of findings.
